# Design and Construction of University Book Layout Based on Text Image Preprocessing Algorithm in Education Metaverse Environment

**DOI:** 10.1155/2022/6219401

**Published:** 2022-09-25

**Authors:** Xinyi Sun

**Affiliations:** DPU Southampton International College, Dalian Polytechnic University, Dalian 116034, China

## Abstract

Books have a significant role in the diffusion of cultural information since they not only carry the weight of cultural inheritance but also serve to preserve historical culture. The major goals of contemporary book layout design are to establish harmony and coherence; maintain overall coordination between the internal and external; and have distinctive, inventive, and modern aesthetic impacts in the context of the educational metacosmos. It is important to emphasize the artistic value and beauty of contemporary books using proper creative language design strategies. The discussion of contemporary book layout design therefore helps to increase understanding of contemporary book layout design. This essay briefly addresses book layout design and examines how books are constructed in colleges and universities. Based on the educational metauniverse environment, it outlines a number of issues that should be taken into account when designing the book's layout. Layout analysis and text image preparation methods are used in modelling. The experimental findings indicate that this algorithm can recognise text regions with an accuracy of 94.8% and a recognition rate of 94.5%, respectively. It is concluded that the method suggested in this work has some reference value for the advancement of university book layout design and can be applied effectively in layout analysis and text typesetting.

## 1. Introduction

With the development of modern science and technology, the concept of science fiction in the 20th century has a realistic basis. With the popularization of new information infrastructure such as cloud computing and big data, the penetration and integration of virtual and reality have been accelerated, making the metauniverse possible. The metauniverse, also known as “mirror world” and “virtual space,” originated from the science fiction Avalanche published in 1992 [1]. In the novel, it reflects the expectation of human beings to break through the limitation of time and space, so that the human body can find a gateway to another sensory experience and form a shared virtual world of “desirable illusion.” In the physical world, people from all over the world can work, live, and communicate with each other through their virtual “avatars” [2]. In 2021, the China metauniverse summit was held, which is also called the first year of the metauniverse. This concept once again triggered a heated debate in the academic community. The metauniverse is technically the integration of information space-time formed by a series of new information technologies [3] such as the Internet and blockchain. From the perspective of industry, education is the main application scenario of metauniverse. This not only reflects that education is positioned as a public welfare undertaking that runs through personal lifelong development but also reflects the integration of technology and education in future education. The education metauniverse is ready to emerge at this moment, which is considered as an effective model to balance technological development and education issues [4]. Compared with the existing virtual reality scene, the education metauniverse has a deeper sociality and is closely related to the attributes and elements of the real society. Therefore, the education metauniverse has a broader and deeper application scenario for the breakthrough of the space-time boundary [5]. This new environment based on the rapid development of computer graphics and computer vision brings people absolute imagination. In the field of education, the metauniverse has attracted the attention of educators because of its combination of virtual reality and digital twins [6].

Design plays a significant role in social culture. It was created and finished with the assistance and constraints of culture, representing the cultural vogue of the day [7]. Culture has an impact on design in every area of life, contributing in and limiting its evolution. An essential element of contemporary college books and modern college book design is the layout. Since the introduction of computer technology into the realm of book layout design, typesetting and manual phototypesetting have been steadily supplanted by computer typesetting, allowing for more design options for book layout [8]. To make the book layout design more vibrant and rich, the designer organically combines classic book design with modern book design against the backdrop of the education metacosmos. Books for universities should have layout designs that stay up with modern developments. The development of books is coordinated with developments in book layout design. Different historical eras' layout designs are highly correlated with their own political economies, levels of productivity, and printing technologies [9]. With the higher and higher aesthetic requirements of the book layout design in colleges and universities, the research and analysis of the book layout in colleges and universities have a very important impact on the aesthetic integrity of the book design. First of all, in the information age, it is very difficult for college students to calm down and concentrate on reading. They pick up a book and generally just skim through it. They make a preliminary judgment on the contents of the book. They can only read it if they think it is necessary. It can be seen that the layout design of the bookcase is directly related to whether a book is attractive to college students and whether it can arouse students' interest in the book [10]. At the same time, if the book layout design of colleges and universities has strong visual impact, attraction, and appeal, it can facilitate the subsequent reading, search and retrieval of book contents for most students, and help them improve the reading effect of books [11]. In a fixed book layout, a unique and distinctive layout style that belongs to the book content is built through layout design, so that it can be accurately integrated with the book content and emotional connotation. The designer needs to make full use of the composition, expression, and application of points, lines, and surfaces in the layout design. Dots, lines, and faces are the basic elements of layout design, the premise of layout design, and the main means of expression of layout design. Based on the education metauniverse, research has great application value and significance for book layout design [12].

Based on this, this paper briefly explores book layout design and evaluates how it is created in colleges and universities using the context of the education metauniverse. The research employs the layout analysis and the text image preprocessing algorithm to represent a number of points that need to be addressed in the book layout design. The algorithm proposed in this paper includes the layout analysis, binarization, and page image deformation. The model is next examined, and it is determined that the layout, design, and creation of university books based on the environment of the education metauniverse have some practical worth. The layout, design, and construction of university textbooks enable readers to enjoy the visual beauty of the text while reading it and fully comprehend its subject matter.

Through the analysis of the background of book layout design and education metauniverse, this paper builds a model of book layout design for colleges and universities based on education metauniverse and analyzes the model. The work and innovation of this paper mainly include the following:

- For the innovation of the topic selection, it combines the education metauniverse environment with the book layout design of colleges and universities and enriches the application theory system of the traditional book layout design. It broadens the application of educational metauniverse in the field of book layout design in colleges and universities. Under the background of education metauniverse environment, it is an innovation to explore the book layout design. By building a model, the important role between the two is obtained, which promotes the common development of education metauniverse and the book layout design of colleges and universities in the future
- In this paper, we use the analysis method of image layout features for reference and apply this method to the traditional content-based image retrieval technology. We propose to extract the row block features from the layout of the text area of the document image and use the extracted row features of the layout as the index items, which can be used for image feature matching and similarity measurement
- An innovative feature matching strategy is put forward in this research. A point in space is created from the acquired line. The position of the point is determined by the starting coordinate of the line, and its brightness is determined by the length of the line. The center point weighted matching algorithm is used in the point matching mode. We use each row's line length as a weight for determining the center point position coordinates and take into account the weighted average of the layout to determine the center point's relative coordinates for global position matching

Starting from the relevant research on the application theory of book layout design, this paper studies how to carry out book layout design and conducts modeling analysis based on the background of education metauniverse environment. The organizational structure of this paper is as follows:

The first section is the introduction, which introduces the research motivation of this paper, expounds the research background and significance of the layout design and construction of university books based on the education metauniverse environment, puts forward the research questions, and gives the research methods. The second section introduces the relevant literature, lists some scholars' research results related to the education metauniverse and book layout design, and puts forward the research methods and ideas of this paper. The third section is the method part. This paper introduces and analyzes the layout design of university books based on the education metauniverse environment and builds the relevant models. The fourth section is the experimental analysis. In this part, experimental verification is carried out on the data set to analyze the effectiveness of the model. The fifth section is the summary and prospect. This section summarizes the full text and explains the layout design of college books based on the education metauniverse environment.

## 2. Related Work

Lunt et al. proposed that decentralisation, multiagent real-time interaction, immersive experience, virtual simulation, and self-satisfaction are among the core phrases of the metaworld. The separation between the actual world and the virtual world must be entirely eliminated in order to achieve smooth docking and complimentary integration of real life and virtual life. As a new way of thinking, the grand scenes produced by the metauniverse, such as decentralisation, decentralisation, real-time interaction between multiple people, and real-time switching between multiple spaces, not only deeply unleash human creativity and initiative but also create a conscious discourse space parallel to the real world without leaving any traces in the virtual world [13]. Ping believes that the wave of metauniverse has promoted the innovation and evolution of all walks of life. Many fields have explored their own advantages and future development directions while conforming to the trend of metauniverse. As the metauniverse of the Internet category, one of its core lies in content creation [14]. McAlpine et al. put forward the idea of continuous promotion of universe technology and metauniverse application. In the future, there will be three major trends in the content production of metauniverse, namely, creative upgrading, computing upgrading, and intelligent upgrading. The framework of education metauniverse is mainly composed of technical support, interactive formats, and rule design [15]. The education metauniverse, according to Guerin et al., is explained as follows: “As participants or organisers of teaching activities, teachers, students, and administrators independently create and participate in teaching activities, immerse themselves in the education meta universe through virtual avatars, and naturally react to the teaching behaviour of the virtual and real worlds. Based on this background, they can break beyond the limits of physical laws and geographical space, and accomplish the two-way transmission of information in the virtual and real world” [16]. Michelle et al. carried out the research from the related design of the table of contents page in the book layout design. Through the study of the aesthetic characteristics of the cover design of popular books, the aesthetic elements of the cover design are analyzed, which are mainly reflected in the beauty of words, colors, and graphics [17]. Binmakhashen and Mahmoud analyzed the elements of text typesetting and expounded the application methods of font typesetting in book layout design. This paper puts forward the language features of form and style in book layout design and analyzes the application of form and style in book layout design. For the shape shaping of art books, including the unity of the function and artistry of book design, the overall beauty and the visual psychology form expression of books, etc. [18]. Vasilopoulos and Kavallieratou believe that the overall layout design of books is a form design based on the basic functions of books and a design of spiritual products with reading as the demand. This basic functional requirement determines the unity and coordination of book form and content. The physical structure, visual characteristics, and external forms of books are all intended to more accurately and effectively convey the theme and content of books, while the content and ideas that are separated from the material carrier and perceptual image cannot be called books [19].

From the research results listed above, we can know that metauniverse, as the hottest technology and thinking concept in recent years, has attracted the attention and discussion of many industries and industry practitioners. The book layout design has always been the content that people attach importance to. How to design the book layout of colleges and universities based on the environment of education metauniverse is very scarce in the current literature, and the relevant theoretical analysis of the combination of the two is also very few. Therefore, this paper will discuss the book layout design based on the education metauniverse environment through consulting relevant documents, which can not only enrich the theoretical system of the education metauniverse but also improve the attention of the school to the book layout design and promote the development of the book layout design field.

## 3. Methodology

### 3.1. Related Concepts of Book Layout Design

The design of all book formats is referred to as “book layout design.” It is a procedure whereby visual components are put together and arranged on a certain layout in a particular way and in accordance with the needs of the book's content and functional system. The high degree of synergy between technology and art is realized by using it as both a vital tool for ensuring the efficient conveyance of information and as a crucial element of contemporary books. Modern layout design has evolved into one of the fundamental abilities required of graphic designers [20]. The book layout design is also the prior art design of the format, font, illustration, cover, and other elements. It is an artistic and reasonable design of the style, structure, level, and illustration of the original on a certain format. Layout design is an interdisciplinary specialty, which involves many disciplines such as aesthetics and colorology. The same book layout design cannot be overlooked. It is an important part of the whole book design. It runs through the whole process of book binding and guides readers to read. Dots, lines, and faces are the basic elements of book layout design and are also the premise of book layout design. Book layout design is also deeply influenced by modern painting. Monterian, a master of Dutch style, used symmetrical, balanced, and straight line composition to directly affect the field of book layout design. In his works, only horizontal lines and vertical lines are used, excluding curves, and simple colors and simple ratios are used on the dividing surface. This color code is based on standardization to obtain the most striking visual effect. Its basic point is not based on the expression of personal emotions, but on the logical and unique arrangement with the layout form, and the mathematical principle is used as the basis of the modeling structure. It is a geometric abstract art that basically excludes the pictorial organization and proportion.

Book layout design is a significant means of information communication. The constant advancement of society, the quickening of life, and the alteration of people's visual habits force designers to update their ideas, give importance to book layout design, take in the best ideas of contemporary design and reposition book layout design, and forge new grounds for the growth of book layout design. The 21st century is an era of information integration, and various knowledge fields are infiltrating each other. It is an important historical mission of modern book layout design to build a communication platform between readers and readers. In fact, the book layout is no longer a simple technical arrangement. The book layout design is a high unity of technology and art, especially the book layout design in the century has been upgraded to a new level. Designers gradually realize the importance and value of book layout design. Using the visual enjoyment brought by the book layout design to the readers to impact people's inner feelings, make the designer and the readers build a bridge, and produce a close communication and emotional shock.

### 3.2. Application Analysis of Book Layout Design Based on Education Metauniverse

As the book is not a static and solidified body, it has a certain relationship with the surrounding environment and belongs to a dynamic life body; therefore, the layout designer should use the art design concept to make the visual beauty of the modern book layout more strong and constantly improve the appeal of the book layout design. With the rapid development of information technology and science, people have higher requirements on the efficiency and ways of obtaining information. Electronic media has rapidly penetrated into people's lives and has quickly replaced paper media with its low cost and high efficiency. Meanwhile, the rise of culture and education has also made people have higher requirements on the aesthetic feeling and function of books. This forces the book designer to say goodbye to the previous single illustration and text design method, but more pursue the expression of culture and emotion, and explore new and original design expression by combining the research and practice of illustration and free layout design. Make the design reach the concept of “design as a person” and conform to the original spirit and the prevailing “craftsman” spirit. In the overall design of modern books, illustration is very important. It is also an important component of the layout design of modern books. It can effectively make up for the lack of text language and enable readers to better grasp the contents of books. The layout design of modern books should truly meet the aesthetic requirements of readers. The form of books should be consistent with the logic of content and have good visual aesthetic impact, so that readers have a new feeling. In modern book layout design, different combinations of fonts, lines, and colors can reflect the characteristics of book layout design. In order to better meet the aesthetic needs of readers, modern book layout designers should effectively combine words, images, and colors to create a good visual image, so that the image thinking of readers can be better extended. In the layout design, the grid system is a very important part. A reasonable and efficient grid system is particularly important for the layout of publications. The depth of the single cell area is consistent with the specific number of lines. The width of the single cell area is the same as the column width. The height and width are indicated by dots or Cicero printing size units. The single cell area is separated by the middle blank area. In the layout design, most of the expected grid areas are either too high or too low. Therefore, it is necessary to fine tune the text lines and grid areas to achieve the effect of mutual agreement and accuracy. Then, the font must be selected to determine whether the font is compatible with the page proportion with aesthetic pleasure. The schematic diagram of the area that text and picture information in the grid may occupy is shown in Figure 1.

In the educational metauniverse environment, the layout design of books is not a “small skill,” but a very important part of the whole book design. Its design runs through the whole process of book design and has a subtle impact on the whole process of readers' reading. Understand some necessary elements of cover layout design. It includes (1) who is the author of the book, (2) what is the theme and main plot of the book, (3) what is the exact size of the book, and what is the size of the envelope and the hinge inside the envelope. In the design of the book cover, it is required to grasp and highlight the content of the book, rationalize the information, sort and arrange the order, and find the visual signs consistent with the content. The idea that form and content should complement one another is crucial when designing the layout of a book's inner pages. Designing forms serves both form and expression. Instead, it emphasizes the content. In order to create the unity of content and form, content determines form, grasps the overall concept, and fully expresses content. It should be obvious that the layout design is not the main objective but rather improved information transmission and viewpoint representation. A well-designed layout has a highly cohesive body that perfectly conveys the material and accurately reflects the designer's design principles. The flexibility of hue is also crucial. Color has a very rich content, is an element that is intimately tied to nature, and may be used to effectively express information. Color analysis is an individualised process. As a result of the profound cultural variations, different people perceive colors in different ways. We must incorporate specific colors into the book layout design in order to better accommodate the requirements of diverse cultures. This will give the colors a particular vibrancy and enable them to show spatial information more effectively. The final stage of the overall design of the book is the adjustment of the overall and partial details of the layout. The processing of the details can enhance the visual rhythm, reading rhythm, and psychological rhythm of the book reading. This stage can reflect the integration and control ability of experience and is also a test of the designer's overall quality, cultivation, vision, and skills.

The picture element in book layout design is the most important element besides text. In addition to the photographic works and art books, the pictures in most books are connected with other pictures or words as an explanation of the auxiliary contents or words. In the layout design of the picture, the size, function, and outline of the picture should be considered. The positional relationship of pictures in the layout, position, size, and proportion of each picture will affect the visual flow of the reader, and it is necessary to consider the shape and content structure of the picture for typesetting design.

### 3.3. The Design and Construction of University Book Layout Based on Education Metauniverse

For the educational metauniverse environment, the layout design of university books includes three parts: layout analysis, layout understanding, and layout reconstruction. The layout analysis operation divides the acquired document image into different regions according to the attributes and marks the types of text, image, table, etc., for each region to prepare for the layout reconstruction operation. In the process of layout understanding, the information obtained through analysis is reprocessed to obtain the logical structure of the document including the logical structure of each area, the hierarchical relationship of the document, and the reading order of the article, so as to obtain the text code that conforms to the original content. The purpose of text image layout segmentation is to obtain relatively independent partitions, i.e., text area, illustration area, and table area, rather than the small connected area of a single character. The method based on connected regions is to find out all connected regions in the image first and then combine them according to the internal spacing, word spacing, and line spacing of characters to form a large connected region. This method is slow. Therefore, before text image segmentation, this paper first fills the text image with text lines, connects the adjacent words and the adjacent lines belonging to the same paragraph, forms a large and relatively independent connected unit, and then performs the next step of segmentation. The schematic diagram of image retrieval principle is shown in Figure 2.

In the feature space, the similarity measure uses the feature vector to describe the attributes of the samples and uses the distance measure to represent the similarity between the features to be matched. The similarity indicates the degree of similarity between the two images compared. The greater the value, the greater the degree of similarity. The distance indicates the degree of discrimination. The greater the value, the greater the difference and the less the similarity. The extracted features are generally represented by vectors, and a vector represents a point in the multidimensional space. The similarity between points can be measured by the distance in the feature space. The text objects of plain text pages have the characteristics of close text spacing and uniform distribution. In view of this characteristic, this paper uses the natural scene based text detection algorithm CTPN and the top-down method to process plain text document images. The flowchart of CTPN algorithm is shown in Figure 3.

CTPN regards the text line as a character sequence instead of a single independent object in general object detection. The relationship between each character image on the same text line can be considered as context, so Bi LSTM layer is added in the training stage to extract the context features of the character sequence, so that the detection model can learn the context statistical features contained in the image. Finally, the text line construction algorithm is used to merge the character sequences. The first step of image analysis is to realize grayscale image analysis. There are only two brightness values of the image: black (pixel is 0) and white (pixel is 255). Let the pixel value of each point of the input image be *f*(*i*, *j*), 255 represent the front scenic spot, and the pixel value of this point of the output image be *h*(*i*, *j*). The expression is as follows:

(1) $$\begin{array}{c} h\left(i,j\right)=\left\{\begin{array}{c} 255,f\left(i,j\right)\leq \text{threshold},\\ 0,\begin{array}{c} f\left(i,j\right),\text{threshold}. \end{array} \end{array}\right. \end{array}$$

First, we define a fuzzy subset that maps from the image *P* to the [0, 1] interval. Professional fuzzy sets are expressed as

(2) $$\begin{array}{c} P=\left\{f\left(x,y\right),\mu_{x}\left(f\left(x,y\right)\right)\right\}. \end{array}$$

We can get the average values *μ*0 and *μ*1 of the color levels of the foreground and background of the image *P* Finally, we can measure the ambiguity according to the Shannon entropy function. The entropy of a fuzzy set *M* is defined as

(3) $$\begin{array}{c} E\left(M\right)=\frac{1}{n\ln2}\underset{k}{\sum }S\left(\mu_{A}\left(x_{k}\right)\right)\;k=1,2,\cdots ,n, \end{array}$$

wherein Shannon function is

(4) $$\begin{array}{c} S\left(\mu_{A}\left(x_{k}\right)\right)=‐\mu_{A}\left(x_{k}\right)\text{In}\left[\mu_{A}\left(x_{k}\right)\right]-\left[1-\mu_{A}\right]\text{In}\left[1-\mu_{A}\left(x_{k}\right)\right]. \end{array}$$

Extended to two-dimensional images, the entropy of images can be expressed as

(5) $$\begin{array}{c} E\left(X\right)=\frac{1}{MNIn2}\underset{i}{\sum }\underset{j}{\sum }S\left(\mu_{A}\left(x_{\text{k}}\right)\right)i=0,1,\cdots M-1,j=0,1\cdots ,N-1. \end{array}$$

In order to determine the connecting line of the text line, it is necessary to find the nearest point to the left and right, respectively, with the reference point as the center. The search method is as follows:

(6) $$\begin{array}{c} W_{\text{left}}=k^{*}\left(D_{x}-S_{x}\right)+\left|D_{y}-S_{y}\right|, \end{array}$$

(7) $$\begin{array}{c} W_{\text{right}}=k^{*}\left(S_{x}-D_{x}\right)+\left|D_{y}-S_{y}\right|, \end{array}$$

where *S* is the current reference point, *D* is the target point, and *k* is the weighting coefficient. Because Chinese and English typesetting are basically horizontal typesetting, and the text lines are horizontal; *k* = 0 is selected here to emphasize the horizontal direction. If the target point with the smallest positive value is selected, it is the left nearest neighbor point or the right nearest neighbor point. The calculation method of the error between the lines of text is as follows:

(8) $$\begin{array}{c} E\left(i,j,k\right)=\overset{R}{\underset{x=L}{\sum }}\left|{\left[C_{j}\left(x\right)-C_{j}\left(x\right)\right]}^{*}K\left(i,j,k\right)+C_{i}\left(x\right)-C_{k}\right|. \end{array}$$

The calculation formula of the best *i*∗ is as follows:

(9) $$\begin{array}{c} i^{*}=\underset{\left(i,j\right)}{\arg\min}\overset{n}{\underset{\begin{array}{c} k=1\\ k\neq i,j \end{array}}{\sum }}E\left(i,j,k\right). \end{array}$$

After two baselines are determined, the image can be restored. Assuming that the point position in the ideal environment is (*x*, *y*) and the actual response in the picture is (*x*_0_, *y*_0_), there is the following corresponding relationship:

(10) $$\begin{array}{c} x^{*}=\int_{0}^{x_{0}}\sqrt{1+{\left[\frac{C_{x0}\left(x\right)}{dx}\right]}^{2}}dx. \end{array}$$

The image to be queried is preprocessed, and necessary denoising and tilt correction are performed on the image. Preprocessing includes feature extraction using images. The preprocessed image is located in the effective area to facilitate operation in the data area. Perform layout analysis on the image to analyze whether the queried image is a plain text image or a document image containing images, tables, etc.; if there is an image or a table area, the nontext area filtering method is used to filter it, and only the text area is retained. The bottom-up analysis method is used to extract the layout line features of the document image, mark the text line of the plain text image, use the ladder interpolation method to fill the step jump in handwriting or English, and then mark the line. After that, the line is abstracted into points in the space, and the center point of the image is found using the weighted average method of the center point, and then, its relative coordinates are calculated. For picture matching based on similarity, the difference energy is used. To find the desired image, perform a search in the image database. Based on this, each feature map is treated as an image in this work. The average filter is applied to all feature maps except the background feature map in order to prevent the diffusion effect of the background white area. Then, the category of the feature map with the highest probability at a specific position on all feature maps is once again selected as the category of the pixel at that location. This technique successfully prevents the occurrence of a tiny region within a larger area that is unrelated to the area's category. In a nutshell, book design includes both the overall design encompassing the content and the surface design. The general layout of books and the rewriting of material information are the current trends in contemporary book design. Each pixel's category will be influenced by the categories of the pixels around it through the overall design, from the inside out. For instance, there is a good chance that a pixel is in a category of text if the pixel category surrounding it is text.

## 4. Result Analysis and Discussion

For the layout design of university books in the educational metauniverse environment, this paper applies the general object detection framework and image semantic segmentation based on pixel level to different data sets. Among them, the ICD AR2017 page object detection data set and the 500 document image data set manually annotated by our laboratory are subject to the page object detection using the anchor box-based detection and regression method, and the ICD AR2009 page object detection evaluation competition data set and the 60 business card image data set manually annotated by our laboratory are subject to the page object detection using the pixel based semantic segmentation method. The experimental data set is shown in Table 1.

At the same time, this paper uses SSD model for testing. Compared with fast RCNN model, the detection results of M APS in the evaluation index of page document objects are lower, mainly because the recall rate is relatively low, but it has a faster detection speed. Therefore, this paper only explores the use of fast RCNN model and makes relevant improvements on the basis of this model. The potential target candidate regions are obtained by traditional image processing methods, and the potential target candidate regions are used as the input of CNN for classification and judgment. The database document images were tested, and the data of 400 images were tested, including four parts of operation results: horizontal and vertical row judgment, title extraction, page number extraction, and column number judgment. Among them, the horizontal and vertical row judgment counts the number of documents in the vertical row, and the column number judgment counts the number of multiple columns (double columns and three columns) as the experimental basis. The experimental data and results are shown in Table 2 and Table 3.

According to the experimental data, the accuracy of simple document test is relatively high in the two tests of horizontal and vertical row judgment and page number extraction. This is because when simple document images are judged horizontally and vertically, the column number dividing line and line spacing are clear, and the title position is obvious when the title is extracted, while nested complex document images are affected by the title and header. At the same time, in the simple document image, the interference of the graph field and the table field is small. Therefore, the accuracy rate of simple document image is relatively high for horizontal and vertical row judgment and page number extraction test. In order to further analyze the design of the book layout, the characteristics of images and characters are further studied. A total of 4950 results were obtained by matching the layout structure of the images in the experiment. The distribution of image energy is shown in Figure 4.

The experimental results obtained using this data show that the difference energy of two different layout structures in these images is about 50 at the minimum and 340 at the maximum. The horizontal axis in Figure 4 shows the number of matching cases of 100 images. The maximum coordinate that can be taken is 4950, and the vertical coordinate is the difference energy corresponding to each matching case. The maximum value is 500. It can be concluded from the Figure 4 that the energy difference is mainly between 50 and 200. The *K*-means clustering results of training sets on different data sets are shown in Figure 5.

The formula objects are grouped into six categories using the two-dimensional *K*-means clustering approach, and the anchor frame scale transformation size and length width ratio are chosen from the centers of each category. The minibatch approach is still used for each image throughout the training. The tags with IOU greater than 0.7 of the real frame are no longer chosen as positive samples in all the generated anchor boxes when picking positive samples. Instead, for each type of item, only the tags in the anchor boxes of the six proportions of the feature map that have IOU values greater than 0.7 of the real frame of the formula and comply to this type's scale transformation are chosen as positive samples.  Figure 6 displays a comparison of recognition rates for several algorithms.

It can be seen from Figure 6 that the recognition rate of the extracted text line region under the algorithm in this paper is the highest, which can reach 94.5%. This method makes the size of the anchor frame transform more targeted for each detected object. However, the premise of this method is that the size and shape of the objects detected in the test set and the training set are similar. In order to further understand the advantages of the algorithm, the running time of different algorithms is compared, and the results are shown in Figure 7.

It can be seen from Figure 7 that the running time of each algorithm changes with the increase of the number of samples. This paper also selects the network selection of the front-end part of fast RCNN and tries to use vgg16 and ResNet101 networks for feature extraction. The comparison results of the accuracy of feature extraction for document images under different algorithms are shown in Figure 8.

ResNet101 is selected for feature extraction of document images with higher accuracy and recall. Therefore, ResNet101 residual network is used as the network for fast RCNN front-end feature extraction in this paper. At the same time, this paper uses SSD general target detection algorithm. After testing, the target detection algorithm is lower than fast RCNN in terms of recall and accuracy, so no further research is conducted. After testing, it is found that the fast RCNN method, which directly uses RESNET to extract features, has a good effect on the detection of tables and pictures, but the detection effect of formulas is poor, the recall rate is relatively low, and many formulas are not detected. According to the results of layout analysis, this paper optimizes the text line extraction algorithm. According to the detection area of the page object, for the specific contract document image recognition task, the extracted form and straight line objects are delined, and the seal object is removed by using the separation color channel, which mainly effectively reduces the information loss of the entire document image and ensures the accuracy of recognition. The experimental results show that the recognition rate of this algorithm for text region can reach 94.5%, and the accuracy rate of feature extraction is 94.8%. It is concluded that the algorithm proposed in this paper can be effectively used in layout analysis and text typesetting.

## 5. Conclusion

Books in colleges and universities are frequently found in three dimensions as a carrier of graphic design against the backdrop of the education metacosmos. Books are beautiful in their size, weight, and volume. A book's level of content is on each page, its flowing aesthetic feeling is created by flipping the pages continuously, and its overall volume reshapes the beauty of three-dimensional space. These three elements all correspond to plane space. As a result, the design of a book's layout has become increasingly crucial. The layout design of contemporary books exhibits modern aesthetic expression in both interior and external forms in accordance with the modern design concept and aesthetic need. According to the background of the education metauniverse, investigating the techniques, tenets, and artistic expression of modern book layout design is helpful for advancing the recognition of modern book layout design and enhancing its artistic and creative qualities. As a result, text image preparation methods and layout analysis are used in this paper's modelling. The algorithms that are suggested in this paper include page image deformation, binarization, and layout analysis. The model is finally examined. The experimental findings indicate that this algorithm can recognise text regions with an accuracy of 94.8% and a recognition rate of 94.5%, respectively. The style, design, and development of university textbooks based on the educational metauniverse environment are found to have some practical applications. The structure and layout of university textbooks enable readers to appreciate the visual appeal of the text while reading and fully comprehend its subject matter.

## Figures and Tables

**Figure 1:** Schematic diagram of area occupation in nine grid.

**Figure 2:** Schematic diagram of image retrieval principle.

**Figure 3:** CTPN algorithm flowchart.

**Figure 4:** Distribution of image energy.

**Figure 5:** *K*-means clustering results of training sets on different data sets.

**Figure 6:** Comparison of extraction and recognition rates under different algorithms.

**Figure 7:** Comparison of running time under different algorithms.

**Figure 8:** Comparison of accuracy of feature extraction of document images.

**Table 1:** Introduction of experimental data set.

Data set	Training set	Test set	Document object	Test method
ICD AR page object detection	1800	950	There are 7 kinds of chart, table, formula, picture, text, separator, and noise	Inspection based on anchor frame Measurement and regression
ICRC laboratory contract documents	500	30	Seal and dividing line	Inspection based on anchor frame
ICD AR page object detection	55	15	Table, image, and public	Measurement and regression
Business card data set	80	30	Formula: 3 kinds in total	Pixel based language

**Table 2:** Statistical results of experimental data.

	Simple document image 0001-0300	Top 100 complex document images
Horizontal and vertical documents (vertical)	26	12
Title	68	29
Page	265	90
Multicolumn	39	1

**Table 3:** System test results.

	Horizontal and vertical documents	Title	Page	Multi column
Total number of false judgments (simple text 200)	12	7	11	5
Accuracy	95.6%	89.4%	85.6%	92.4%
Total number of false judgments (complex text 200)	4	2	6	1
Accuracy	84.6%	78.6%	92.1%	98.6%

## Data Availability

The data used to support the findings of this study are available from the corresponding author upon request.
